This article has been retracted.

# Clinical Effect and Safety Analysis of 2.5 *μ*g/kg DEX Nasal Drop in Child Undergoing Ultrasound Examination

**DOI:** 10.1155/2022/3486313

**Published:** 2022-04-12

**Authors:** Haiya Tu, Jing Lin, Jinjin Huang

**Affiliations:** ^1^The Department of Anesthesiology, Children's Hospital of Zhejiang University School of Medicine, Hangzhou 310051, China; ^2^The Department of Anesthesiology, the First Affiliated Hospital of Wenzhou Medical University, Wenzhou 325099, China

## Abstract

In order to meta-analyze the clinical effect and safety of dexmedetomidine (DEX) intranasal sedation in child ultrasound examination, literature retrieval is carried out in Wanfang Medicine, PubMed database, domestic medical research journals. The relevant medical information literature on clinical effects and safety are analyzed by using Rev Man 5.2 software. The retrieved literature is screened according to the research object, method, disease type and other criteria. The results of meta-analysis show that dexmedetomidine intranasal sedation is applied to child undergoing ultrasound examination, and the SPO2 and sedation time are significantly higher than those in the conventional sedation group (*P* < 0.05). The time/score is significantly lower than that in the conventional sedation group (*P* < 0.05), and the incidence of adverse reactions in the dexmedetomidine intranasal sedation group is significantly lower than that in the conventional sedation group (*P* < 0.05).

## 1. Introduction

For young children, during the clinical ultrasound examination, the child needs to be kept in an absolute still state for at least 10 minutes, so the child needs to be sedated [1]. The most commonly used sedative drugs include midazolam, chloral hydrate, etc., but the sedative effect of these drugs is not significant, and they can also cause adverse reactions such as spasm and respiratory depression in children, which pose a serious threat to the safety of children [2]. Dexmedetomidine hydrochloride (DEX) is an *α*2 receptor agonist with the advantages of potency and high selectivity. At the same time, it can produce a sedative effect like normal sleep. The sedation occurs faster and does not inhibit the breathing of the body. It is a sedative with good effect and high safety [3]. Relevant studies have pointed out that dexmedetomidine can be used as a preoperative or pre-examination sedative drug [4], but the effect evaluation of this drug and other related sedative drugs is not yet comprehensive. The relevant literature applied during the examination will further evaluate the clinical effect and safety effect of DEX on infant ultrasound examination based on the support of the literature, and provide reference data for the follow-up in-depth research and clinical promotion of DEX.

The type of research and experiment is randomized controlled trials (RCT). The search direction is the clinical effect and safety of DEX on child ultrasound examination. The search keywords include dexmedetomidine (DEX), ultrasound examination, child, blood oxygen saturation (SpO2), sedation time, recovery time/Scores and incidences of adverse reactions are searched in domestic and foreign literature databases such as Wanfang Medicine, CNKI, VIP, and PubMed for literature within 5 years that matched the search keywords and search directions, and contacted medical research experts in related fields to obtain reference information. When the data is missing or the results are unclear, the original author should be contacted immediately to correct and improve the literature data in a timely manner. Understand the research ideas and content according to the literature abstract, and strictly screen the literature that meets the relevant conditions of DEX, child, ultrasonography, etc. The research must pass the review and approval of the relevant institutions. The relevant operations of the research are completed by professionals and there are no obvious mistakes. Read the literature screened for the first time is screened out with inconsistencies in research methods, duplication of content, and imprecise operations. On the basis of the included literature, RevMan 5.2 software is used for meta-analysis.

All patients in the study meet the age standard of 3–10 years old; (2) the intervention measures are dexmedetomidine sedation and conventional sedation mode, and the differences in the indicators after intervention are compared between the two groups; (3) the research objectives are not selected. Restrictions such as nationality, age, gender, salary, and race are set; (4) loss to follow-up rate is less than 20% during follow-up; (5) research must be reviewed and approved by relevant institutions; (6) literature has been published within the past 10 years; (7) the original clinical data are complete or contact the original author to improve the data; (8) there is no operational error during the study; (9) except for the study sample size, there is no difference in other variables.

The rest of this paper is organized as follows: Section 2 discusses related work, followed by proposed literature search algorithm in Section 3. Meta-analysis results of the effect of dexmedetomidine intranasal sedation is discussed in Section 4.  Section 5 shows clinical tests and data analysis. Finally, Section 6 concludes the paper with summary and future research directions.

## 2. Related Work

The patients included in the study do not meet the age standard; (2) animal experiments; (3) not related to the research topic; (4) review, meta, case report, conference abstract; (5) severe cognitive impairment and mental illness disease; (6) withdrawal or interruption of follow-up during follow-up, resulting in a loss of follow-up rate of ≥20%; (7) no intervention with dexmedetomidine sedation.

Blood oxygen saturation (SPO2), sedation time (sedation time), Wake Time/Score and the incidence of adverse reactions after dexmedetomidine sedation and conventional sedation mode intervention.

For randomized controlled studies, the quality of the literature is evaluated using the modified Jadad rating scale, which has a total score of 7, with 1–3 as low quality and 4–7 as high quality. For cohort studies, the Chinese version of the modified NOS scale is used to evaluate the quality of the literature. The scale has a total score of 10, with<5 as low quality and ≥5 as high quality.

The research data are entered into RevMan5.2 statistical software for analysis. Enumeration data are expressed as risk ratio (RR), and weighted mean difference (WMD) or standard mean difference (SMD) are selected as analytical statistic. All effect sizes are expressed with 95%confidence interval (CI). Heterogeneity between the results of each study is tested by Chi2. When the heterogeneity among the studies satisfies *P* < 0.1 and I2 ≥ 50%, which is statistically significant, the source of this property is analyzed by subgroup or sensitivity; when the heterogeneity among the studies satisfies *P* > 0.1, when I2 < 50%, the heterogeneity is not statistically significant, and the Meta-analysis is carried out with a fixed-effect model. When the source of heterogeneity is unclear, a random-effects model is used in the analysis, and descriptive analysis is used to analyze obvious clinical and methodological heterogeneity.

## 3. Our Proposed Literature Search Algorithm

After searching Chinese and English literature databases such as Wanfang, CNKI and PubMed according to the research direction, keywords and restrictions, a total of 300 literature are searched and screened according to the inclusion and exclusion criteria, and finally 7 literature are included, of which 2 are English literature, 5 Chinese literature, the specific retrieval process is attached in Figure 1. There are 2 low quality and 5 high quality articles in the included studies.  Table 1 shows the basic characteristics and quality assessment results of the included studies. Figure 1 is flowchart of literature selection.  Table 1 is basic characteristics of literature.

A total of 7 papers are included, all of which contained the word “random,” and all of them explained the research methods in detail, and the research methods are in line with the standards [12]. There are no operational errors in the research. The results of publication bias assessment showed that the risk of bias of the included studies is low.  Figure 2 is clinical efficacy and safety of dexmedetomidine intranasal sedation in child undergoing ultrasonography.

## 4. Meta-Analysis Results of the Effect of Dexmedetomidine Intranasal Sedation

A total of 5 literature are included, and the results of the heterogeneity test showed that there is heterogeneity among the literature (*I*2 = 79.0%, *P* = 0.0009). Using a random effect model analysis, the SPO2 of the dexmedetomidine nasal sedation group is significantly higher than that of the routine In the sedation group, the difference is statistically significant after the combined studies (*RR*: 2.37, 95% *CI*: (1.04, 3.70), *P* = 0.0005). Nasal sedation with dexmedetomidine is thought to increase infant SPO2 levels.  Figure 3 is forest plot of the effect of dexmedetomidine intranasal sedation on SPO2 in child undergoing ultrasonography.  Figure 4 is funnel plot of the effect of dexmedetomidine intranasal sedation on SPO2 in child undergoing ultrasonography.

A total of 6 literature are included, and the results of heterogeneity test showed that there is heterogeneity among literature (*I2* = 98.0%, *P* < 0.00001). Using random effect model analysis, the sedation time of dexmedetomidine nasal sedation group is longer than that of conventional sedation. The group is higher, and the difference is statistically significant after the combined studies [*RR*: 3.53, 95% *CI*: (1.25, 5.81), *P* < 0.00001]. Nasal sedation with dexmedetomidine may be considered to increase the duration of sedation in child examined on ultrasonography.  Figure 5 is forest plot of the effect of dexmedetomidine intranasal sedation on sedation time in child undergoing ultrasonography.  Figure 6 is funnel plot of the effect of dexmedetomidine intranasal sedation on sedation time in child undergoing ultrasonography.

## 5. Experimental Tests and Data Analysis

A total of 3 literature are included, and the heterogeneity test results showed that there is heterogeneity among the literature (*I2* = 92.0%, *P* < 0.00001). The random effect model is used to analyze the recovery time/score ratio of the dexmedetomidine nasal sedation group. Routine sedation group is lower, and the difference is statistically significant after the combined studies (*RR*: −13.21, 95% *CI*: (−17.17, −9.26), *P* < 0.00001). Nasal sedation with dexmedetomidine is thought to improve infant recovery time/score.  Figure 7 is forest plot of the effect of dexmedetomidine intranasal sedation on wake-up time/score in child undergoing ultrasonography.  Figure 8 is funnel plot of the effect of dexmedetomidine intranasal sedation on wake-up time/score in child undergoing ultrasonography.

A total of 6 studies are included. The results of the heterogeneity test showed that there is no heterogeneity among the literature (*I2* = 0%, *P* = .49), and the heterogeneity is not statistically significant. The adverse reactions in the fixed nasal sedation group are lower than those in the conventional sedation group, and the difference is statistically significant after the combined studies (*RR*: .24, 95% *CI*: (0.13, 0.46), *P* < 0.0001). It can be considered that intranasal sedation with dexmedetomidine can reduce the incidence of adverse reactions in child and young children during ultrasound examination.  Figure 9 is forest plot of the effects of medetomidine intranasal sedation on adverse reactions in child undergoing ultrasonography.  Figure 10 is funnel plot of the effect of medetomidine intranasal sedation on adverse reactions in child undergoing ultrasonography.

After excluding and merging the data of the included 7 references, the results showed that there is no significant change in the Meta results of the 4 indicators, indicating that there is no obvious heterogeneity among the 7 included references, so it had a high reference value.  Table 2 is sensitivity analysis of literature.

With the progress and development of medicine, various sedative drugs have been widely used in clinical practice, but the defects of some common sedative drugs limit their clinical application, such as the application of ketamine, especially in large doses The application may cause severe malignant and vomiting in the body, and even nystagmus and hallucinations in severe cases; and the application of chloral hydrate will significantly reduce the predictability of the body's onset of action, and it will play a role in the human body for a long time, which can easily lead to respiratory depression, arrhythmia, and even permanent nerve damage; midazolam is a relatively common sedative drug, but it plays a role in human nerves, causing restlessness, cognitive impairment. Therefore, the above-mentioned conventional sedative drugs are not ideal drugs for clinical sedation, especially for child who are not fully developed. Dexmedetomidine is a new and highly selective *α*2-receptor agonist. It has significant effects whether it is sedative or analgesic. It mainly inhibits the body's sympathetic nerves and stabilizes hemodynamics. At the same time, the secretion of glands can be inhibited to avoid the occurrence of respiratory depression.

In this paper, after applying routine sedation and dexmedetomidine intranasal sedation to child undergoing ultrasound examination, the results showed that in terms of efficacy, dexmedetomidine intranasal sedation is applied in child undergoing ultrasound examination, and its SPO2 and sedation. The time is significantly higher than that of the conventional sedation group, and there is still a particularly large difference between them (*P* < 0.05). There is still a particularly large difference (*P* < 0.05); indicating that the induction time of dexmedetomidine instillation of nasal sedation is shorter and the patient is easy to accept. In terms of safety, the incidence of adverse reactions in the dexmedetomidine nasal sedation group is significantly lower than that in the conventional sedation group, and there is still a particularly large difference between them (*P* < 0.05). Nasal administration is a noninvasive route of administration that does not cause discomfort and is easily accepted by children. And compared with other conventional methods, intranasal administration is a noninvasive and simple method, which can significantly improve compliance and tolerance. The lymphatic system and capillary network of dexmedetomidine, the drug can be absorbed and sent to the whole body during the process, and the mucosa connected with the central nervous system can send the drug to the brain, so the effect of dexmedetomidine intranasal administration is faster. And it will not affect the body's stomach or liver.

At present, the application of dexmedetomidine intranasal sedation for child ultrasound examination is still in the stage of extensive research. Relevant researches on the mechanism of action and prevention of complications have achieved great results, laying a research sample basis for meta-analysis. In the literature related to ultrasound examination of child, there are few types that consider the efficacy and safety of treatment, and the results of specific related experiments are not convincing due to errors and chance. In this study, the sample size is increased in the meta-analysis, and the heterogeneity among the studies is reduced. The quantitative analysis of the nasal sedation effect of dexmedetomidine can make the results more scientific and reliable. Although this research has achieved certain results, there are still limitations. Because this research has been screened with reference to specific criteria, a total of 7 papers have been included, and the scope of the collection is the Wanfang database, various medical Chinese journals and other related research topics in the past 5 years. On the whole, the scope of selection is relatively small, and the countries selected for the literature are relatively limited, which may affect the research results and cause errors. In future research, the scope of literature search should be expanded to ensure that meta-analysis is carried out on the basis of sufficient sample size to obtain higher-quality information data, so as to improve the reliability of meta-analysis results and make them more convincing.

## 6. Conclusion

In order to meta-analyze the clinical effect and safety of dexmedetomidine(DEX)intranasal sedation in child ultrasound examination, Literature retrieval is carried out in Wanfang Medicine, PubMed database, domestic medical research journals and biomedical literature and other medical databases. In conclusion, the meta-analysis of 7 literature-controlled trials in this systematic review shows that the results are relatively stable and reliable, indicating that the application of dexmedetomidine intranasal sedation during child ultrasound examination is more effective and safe, which is beneficial for child ultrasound examination. Sedation during the examination can reduce the incidence of adverse reactions, and provide a more valuable reference for the research and application of sedation during infant ultrasound examination.

## Figures and Tables

**Figure 1:** Flowchart of literature selection.

**Figure 2:** Clinical efficacy and safety of dexmedetomidine intranasal sedation in child undergoing ultrasonography.

**Figure 3:** Forest plot of the effect of dexmedetomidine intranasal sedation on SPO2 in child undergoing ultrasonography.

**Figure 4:** Funnel plot of the effect of dexmedetomidine intranasal sedation on SPO2 in child undergoing ultrasonography.

**Figure 5:** Forest plot of the effect of dexmedetomidine intranasal sedation on sedation time in child undergoing ultrasonography.

**Figure 6:** Funnel plot of the effect of dexmedetomidine intranasal sedation on sedation time in child undergoing ultrasonography.

**Figure 7:** Forest plot of the effect of dexmedetomidine intranasal sedation on wake-up time/score in child undergoing ultrasonography.

**Figure 8:** Funnel plot of the effect of dexmedetomidine intranasal sedation on wake-up time/score in child undergoing ultrasonography.

**Figure 9:** Forest plot of the effects of medetomidine intranasal sedation on adverse reactions in child undergoing ultrasonography.

**Figure 10:** Funnel plot of the effect of medetomidine intranasal sedation on adverse reactions in child undergoing ultrasonography.

**Table 1:** Basic characteristics of literature.

author	Year of publication	Outcomes	Quality score
Huang jiajia [5]	2021	(1), (2), (3), (4)	6
Gao yi [6]	2021	(2), (3), (4)	5
Yang haikou [7]	2021	(1), (2), (3), (4)	7
Yao shengjie[8]	2020	(1), (2), (4)	6
Wu guanghua[9]	2021	(1), (3), (4)	5
Jumle a [10]	2020	(1)	4
Ama *E* H [11]	2017	(3), (4)	3

**Table 2:** Sensitivity analysis of literature.

ending	*RR*/WMD 95% *CI*	*P*	*I2*
SPO2	2.37 (1.04, 3.70)	0.0005	79.0
Overall (5)			
Sensitivity analysis			
Sedation time	3.53 (1.25, 5.81)	<0.00001	98.0
Overall (3)			
Sensitivity analysis			
Wake time/score	-13.21 (-17.17, -9.26)	<0.00001	92.0
Overall (4)			
Sensitivity analysis			
The incidence of adverse reactions	0.24 (0.13, 0.46)	0.0001	0.0
Overall (3)			
Sensitivity analysis			

## Data Availability

The simulation experiment data used to support the findings of this study are available from the corresponding author upon request.
